The article "Efficacy of Sequential Capecitabine on Adjuvant Chemotherapy of Triple-Negative Breast Cancer" was published in 2022. Journal: J Healthc Eng.

# Efficacy of Sequential Capecitabine on Adjuvant Chemotherapy of Triple-Negative Breast Cancer

**DOI:** 10.1155/2022/7430775

**Published:** 2022-02-28

**Authors:** Xun Xi, Xingwei Huang, Huozhong Yuan, Jun Ni, Fulan Yang

**Affiliations:** Department of Thyroid and Breast Surgery, The People's Hospital of Ganzhou, Ganzhou Affiliated Hospital of Nanchang University, Ganzhou 341000, Jiangxi Province, China

## Abstract

This paper aims to evaluate the efficacy of capecitabine as extended adjuvant treatment after anthracycline and paclitaxel combined adjuvant chemotherapy for women with early triple-negative breast cancer (TNBC). The patients with early TNBC were randomly assigned to capecitabine sequential treatment for 4 cycles and without any sequential treatment in the control group after anthracycline and paclitaxel combined adjuvant chemotherapy. The primary end point was disease-free survival (DFS). The secondary end point was overall survival (OS). One hundred patients were enrolled in this study between June 2013 and February 2015. Median age was 49 years ranging from 25 to 66 years and treatment was well tolerance. The median follow-up time after random allocation was 58 months (range: 11–62 months). There was no significant difference in DFS and OS between the two groups (hazard ratio (HR) of DFS was 0.50; 95% CI, 0.24–1.05; *P*=0.066). Our study shows that although the addition of four cycles capecitabine after anthracycline and paclitaxel combining adjuvant chemotherapy does not improve DFS and OS, but the trend of DFS is improved. The possible reason is that the four-cycle treatment of capecitabine is not enough, and another possible reason is that the number of cases is not enough.

## 1. Introduction

Triple-negative breast cancer (TNBC) is a heterogeneous breast cancer subtype that is a complex and aggressive breast cancer with a poor prognosis. It accounts for approximately 10–18% of breast cancers. Up to now, there are abundant trials for the therapy of TNBC, but the optimal regimen is ambiguous. Although many trials showed that it could benefit from adjuvant anthracyclines and/or paclitaxels [1, 2], however, even with this relatively effective chemotherapy, the 10-year recurrence rate of early TNBC is still close to 20–40% [3]. There were other trials which suggested that the addition of other new agents including capecitabine, platinum-based agents, and ixabepilone could improve the prognosis.

Capecitabine (Xeloda) is an oral fluorouracil prodrug. During its ingestion in the liver and in tumor cells that contain thymidine phosphorylase, it can be converted to fluorouracil, potentially enhancing intratumoral concentrations of fluorouracil [4]. In the past, several prospective clinical trials have suggested that capecitabine improves the rate of progression-free survival and prognosis in the rescue treatment of metastatic breast cancer who have previously received anthracycline and paclitaxel [5, 6]. In recent years, some studies about capecitabine for therapy were also carried out in (neo)adjuvant therapy. They showed that addition of capecitabine to TNBC could improve prognosis, either combination therapy or sequential therapy after neoadjuvant [3]. However, some conclusions were conflicting.

The article "Efficacy of Sequential Capecitabine on Adjuvant Chemotherapy of Triple-Negative Breast Cancer" was published in 2022. Journal: J Healthc Eng.

At present, there is no study about sequential capecitabine after anthracycline and paclitaxel combined adjuvant therapy. Therefore, we decided to carry out a trial that received capecitabine sequential treatment for 4 cycles after anthracycline and paclitaxel combined adjuvant therapy in the early stage TNBC.

## 2. The Proposed Methods

This is a prospective randomized phase II study in the People's Hospital of Ganzhou, Jiangxi Province, China. 100 eligible patients were enrolled between June 2013 and February 2015 who had completed anthracycline and paclitaxel combined adjuvant therapy. Eligible patients were randomly allocated in a 1 : 1 ratio to receive either capecitabine (experimental group) or no therapy (control group). Patients assigned to the experimental group received capecitabine 1000 mg/m^2^ PO twice daily (every 12 h, and taken 30 min after meals) on days 1 to 14 of the 21-day cycle for four cycles. Patients of the two groups received postoperative radiotherapy after chemotherapy if they needed.

### 2.1. Inclusion Criteria

(a) Early breast cancer with positive axillary lymph nodes or node-negative cancer with tumor diameter ≥20 mm. (b) The primary tumor was diagnosed as triple-negative breast cancer which was absence of amplification of estrogen receptor (ER), progesterone receptor (PR), and human epidermal growth factor receptor 2 (HER2) by immunohistochemistry (IHC). The cell nuclear staining ＜1% of ER and PR was regarded negative, and HER2 assessment was scored from 0 to 3 in immunohistochemistry. HER2, 3+ was defined as positive, and 0 or 1+ as negative. If HER2 was scored at 2+, we should reassess it by fluorescence in situ hybridization (FISH). The FISH was performed according to the ASCO/CAP guidelines [7]. (c) The adjuvant chemotherapy included anthracycline and paclitaxel. (d) The time interval between postoperative adjuvant chemotherapy and the date of randomization was less than 4 weeks. (e) Hemoglobin level >10 g/dl, leukocyte count >4000/*μ*l, absolute neutrophil count >1500/*μ*l, platelet count >100000/*μ*l, bilirubin <1.5 upper normal limit (UNL), aspartate aminotransferase (AST)/alanine aminotransferase (ALT) <2.5, and creatinine <1.5 UNL. (f) World Health Organization performance status less than 2. (g) All patients who received capecitabine should sign informed consent forms.

The article "Efficacy of Sequential Capecitabine on Adjuvant Chemotherapy of Triple-Negative Breast Cancer" was published in 2022. Journal: J Healthc Eng.

### 2.2. Exclusion Criteria

(a) Advanced breast cancer. (b) With neoadjuvant therapy including chemotherapy, radiotherapy, and endocrine therapy. (c) Bilateral breast cancer, inflammatory breast cancer, or carcinoma in situ.

### 2.3. Follow-Up

We followed up the enrolled patients every 3 months. The primary end point of this study was disease-free survival, which was defined as the time from randomization to recurrence, the development of a second cancer, or death from any cause. The secondary end point was overall survival, which was defined as the time from randomization to death from any cause.

### 2.4. Statistical Analysis

Using the Kaplan–Meier method and the unadjusted Cox proportional hazards model to compare disease-free survival and overall survival between the two groups and to calculate the HRs and their 95% confidence intervals (CIs), statistical analyses were performed with SPSS (version 25, IBM) software.

## 3. Experimental Results

The total number of patients in both groups was 50. The mean age of the trial group was (46.3 ± 7.4 years), tumor diameter (26.8 ± 4.9 mm), and positive lymph nodes 37 (74%). Mean age (46.9 ± 6.1 years), tumor size (26.6 ± 5.0 mm), and positive lymph nodes 34 (68%) in the control group. The disease characteristics of the patients are presented in Table 1. There was no statistical difference for the two groups.

The median follow-up time of the patients in the group was 58 months (range: 11–62 months), one lost to follow-up in the trial group and the same in the control group. Of the 49 evaluable patients in the trial group, 11 had recurrence (22.4%), of which 3 had local regional recurrence and 8 had distant metastasis. While 19 of the 49 evaluable patients in the control group (38.8%) had recurrence, of which 5 had local regional recurrence and 14 had distant metastasis. In the evaluable patients of both groups, 9 (16.3%) died in the trial group and 14 (28.3%) in the control group. Both groups of deaths were all breast cancer-specific mortality. DFS differences between the two groups were not statistically significant (HR, 0.50; 95% CI, 0.24–1.05; *P*=0.066) in Figure 1. There was no significant difference in OS between the two groups (HR, 0.50; 95% CI, 0.21–1.19; *P*=0.12) in Figure 2.

## 4. The Result Discussion

For hormone receptor and/or HER2 positive breast cancer patients, we can give endocrine therapy and targeted therapy following chemotherapy and they can improve DFS and OS. Nevertheless, for TNBC, which is a complex and aggressive breast cancer with a poor prognosis, we still do not have an optimal protocol. Previous studies with the addition of paclitaxel on the basis of anthracyclines can make an absolute benefit of about 6–7% in 5–10 years of DFS and OS [8, 9]. Can TNBC benefit from addition of another regimen? We can try to consider the following aspects [10, 11]: (a) addition of drugs in adjuvant therapy [12], (b) duration of adjuvant chemotherapy [2], (c) increasing the dose intensity of cytotoxic therapy by shortening the intervals between cycles [13].

The article "Efficacy of Sequential Capecitabine on Adjuvant Chemotherapy of Triple-Negative Breast Cancer" was published in 2022. Journal: J Healthc Eng.

FinXX trials conducted in Finland and Sweden compared the recurrence-free survival (RFS) and survival between groups receiving 3 cycles of docetaxel followed by 3 cycles of cyclophosphamide, epirubicin, and fluorouracil (*T* + CEF) and received 3 cycles of docetaxel plus capecitabine followed by 3 cycles of cyclophosphamide, epirubicin, and capecitabine (TX + CEX) in the invasive breast cancer patients with positive regional lymph nodes or node-negative cancer with tumor diameter ≥20 mm and negative progesterone receptor expression (<10% of cancer cell nuclei stained positive). This trial suggested that capecitabine administration with docetaxel, epirubicin, and cyclophosphamide did not prolong RFS or overall survival compared with a regimen that contained only standard agents (hazard ratio (HR), 0.88; 95% CI, 0.71–1.08; *P*=0.23; and HR, 0.84; 95% CI, 0.66–1.07; *P*=0.15, respectively). Patients with TNBC had favorable survival outcomes when treated with the capecitabine containing regimen in an exploratory subgroup analysis (HR, 0.53; 95% CI, 0.31–0.92; *P*=0.02) [14]. Similar to FinXX trial, 585 early TNBC patients were randomly assigned to T-CEF or TX-CEX in China. After a median follow-up time of 30 months, there was no significant difference in the primary end point (DFS) between the two groups. A total of 2611 patients were enrolled in the US Oncology NO1062 trial [15]. The patients were randomly assigned to receive 4 cycles of AC followed by 4 cycles of docetaxel (AC-T) or 4 cycles of AC followed by 4 cycles of TX (AC-TX), about 70% of the patients were lymph node positive. The study found that there was no significant difference in DFS (HR = 0.81; 95% CI, 0.57–1.15) between the two groups, while there was a significant increase in OS (HR = 0.62; 95% CI, 0.41–0.94) in favor of AC-TX for TNBC subgroup. Our study was sequential capecitabine after adjuvant chemotherapy rather than combination chemotherapy.

CIBOMA/2004–01/GEICAM/2003–11 trials evaluated the efficacy of adjuvant capecitabine in operable TNBC patients with lymph node-positive or node-negative with tumor diameter ≥10 mm after standard anthracycline and/or taxane containing (neo)adjuvant chemotherapy. They were randomized to receive eight cycles of capecitabine (1000 mg/m^2^ bid, d1-14 q21 d) or observation. The primary end point is disease-free survival (DFS). This study failed to show a statistically significant increase in DFS by adding extended capecitabine to standard (neo)adjuvant chemotherapy in patients with early TNBC (HR = 0.82; 95% CI, 0.63–1.06; *P*=0.136). In addition, there was no statistically significant difference in OS between the study arms (unadjusted HR, 0.92; 95% CI, 0.66–1.28; *P*=0.623) [16]. Although in this study, its exploratory subgroup analysis for DFS included capecitabine sequential adjuvant chemotherapy, but the adjuvant chemotherapy included anthracycline and/or taxane regimens rather than anthracycline and taxane. Our study only received the combination adjuvant chemotherapy agents of anthracycline and taxanes.

The article "Efficacy of Sequential Capecitabine on Adjuvant Chemotherapy of Triple-Negative Breast Cancer" was published in 2022. Journal: J Healthc Eng.

While in the CREATE-X study, its trial design was that patients with residual invasive breast cancer components after standard neoadjuvant chemotherapy which used anthracycline and/or taxane regimens were assigned into the capecitabine treatment group and control group, and the patient of this study was HER2-negative including hormone receptor positive patients. Among patients with TNBC, the rate of DFS was 69.8% in the capecitabine group versus 56.1% in the control group (HR for recurrence, second cancer, or death, 0.58; 95% CI, 0.39–0.87), and the overall survival rate was 78.8% versus 70.3% (HR for death, 0.52; 95% CI, 0.30–0.90) [17]. Our study only included the adjuvant chemotherapy but not neoadjuvant.

Thus far, some studies evaluated metronomic capecitabine as an extended adjuvant therapy in TNBC patients. In 2015, Alagizy et al. carried out a prospective phase II study which recruited 41 patients diagnosed with TNBC who had completed 6 cycles of FEC adjuvant chemotherapy ± postoperative radiotherapy chemotherapy. They received capecitabine 500 mg PO twice daily (once every 12 hours, half an hour after meal) and continuously for six months as an extended adjuvant therapy. The study showed that the tolerance was well with no level 3 or level 4 toxicity or life-threatening adverse events. In the study, only 6 (15%) recurrent events were occurred. The mean DFS was 42.4 months and the mean OS was 44.3 months. Although there is no control group in this study, it also suggested the feasibility of metronomic capecitabine treatment [12]. Another phase III randomized study, SYSUCC-001, was also to evaluate the efficacy of capecitabine metronomic chemotherapy for 1 year (650 mg/m^2^, PO, twice a day) after standard adjuvant chemotherapy. The results of this study have not been released.

The article "Efficacy of Sequential Capecitabine on Adjuvant Chemotherapy of Triple-Negative Breast Cancer" was published in 2022. Journal: J Healthc Eng.

The possible reasons for the effectiveness of capecitabine in the treatment of TNBC are still uncertain. The possible reasons may be that capecitabine is administered every day and the addition of capecitabine in a standard chemotherapy regimen may lead to (a) the enhancement of chemotherapy drugs, (b) the longer exposure of tumor cells to fluorouracil compared with intravenous injection of fluorouracil that has a short half-life in plasma [18–20], and (c) the higher concentration of fluorouracil in tumor cells.

## 5. Conclusion

This paper aims to evaluate the efficacy of capecitabine as extended adjuvant treatment after anthracycline and paclitaxel combined adjuvant chemotherapy for women with early triple-negative breast cancer. Our paper shows that the DFS and OS have not been improved in addition, four cycles of sequential capecitabine after standard anthracycline and taxane regimens containing adjuvant chemotherapy, but DFS has a trend of improvement, which may be caused by the insufficient treatment cycles of capecitabine only four cycles, the insufficient number of cases, or the insufficient follow-up.

## Figures and Tables

**Figure 1:** DFS indicates disease-free survival; HR, hazard ratio; group control, without any sequential treatment after anthracycline and paclitaxel combined adjuvant chemotherapy.

**Figure 2:** OS indicates overall survival; HR, hazard ratio; group capecitabine with capecitabine sequential treatment for 4 cycles after anthracycline and paclitaxel combined adjuvant chemotherapy.

**Table 1:** The characteristics of patients.

Characteristics	Capecitabine N (%)	Control N (%)	Statistics	*P* value
Median age (y)	46.3 ± 7.4	46.9 ± 6.1	*T*-test	0.33
Median tumor diameter (mm)	26.8 ± 4.9	26.6 ± 5.0	*T*-test	0.91
Axillary nodal status			Chi-square	0.79
pN0	13(26%)	16(32%)		
pN1	31(62%)	29(58%)		
pN2	6(12%)	5(10%)		
Histological grade			Chi-square	0.81
2	40(80%)	38(76%)		
3	10(20%)	12(24%)		
Stage			Chi-square	0.94
IIA	15(30%)	16(32%)		
IIB	29(58%)	29(58%)		
IIIA	6(12%)	5(10%)		

## Data Availability

The data used to support the findings of this study are available from the corresponding author upon request.
